# A Massage Area Positioning Algorithm for Intelligent Massage System

**DOI:** 10.1155/2022/7678516

**Published:** 2022-08-04

**Authors:** Liran Zhou, Zhiquan Feng, Zeyuan Cai, Xiaohui Yang, Changsheng Ai, Haiyan Shao

**Affiliations:** ^1^School of Information Science and Engineering, University of Jinan, Jinan 250022, China; ^2^Shandong Provincial Key Laboratory of Network Based Intelligent Computing, Jinan 250022, China; ^3^State Key Laboratory of High-end Server & Storage Technology, Jinan 250002, China; ^4^School of Mechanical Engineering, University of Jinan, Jinan 250022, China

## Abstract

A growing number of studies have been conducted over the past few years on the positioning of daily massage robots. However, most methods used for research have low interactivity, and a systematic method should be designed for accurate and intelligent positioning, thus compromising usability and user experience. In this study, a massage positioning algorithm with online learning capabilities is presented. The algorithm has the following main innovations: (1) autonomous massage localization can be achieved by gaining insights into natural human-machine interaction behavior and (2) online learning of user massage habits can be achieved by integrating recursive Bayesian ideas. As revealed by the experimental results, combining natural human-computer interaction and online learning with massage positioning is capable of helping people get rid of positioning aids, reducing their psychological and cognitive load, and achieving a more desirable positioning effect. Furthermore, the results of the analysis of user evaluations further verify the effectiveness of the algorithm.

## 1. Introduction

As health care has aroused the rising attention of people, it has become a trend to integrate intelligent massage robots into people's daily lives to help them achieve massage and relaxation anytime and anywhere. Massage positioning is recognized as the first task of an intelligent massage robot, and numerous existing research results have been achieved relating to massage positioning.

Three main types of massage systems have been used on the market over the past few years. The first one is the larger massage chair, which is the most common and requires the operation of a remote control or control panel to give the massage positioning instructions. This positioning mode of operation, however, is not friendly to the elderly and has a rigid division of massage areas. The second type refers to a small regional massager (e.g., a neck massager). The above type of massager is focused and can only be applied in one area. The third type refers to the professional type massage robot arm, which is primarily employed in professional massage hospitals or massage shops. The user should lie in a fixed position after completing the diagnosis, and the massage position is set by the professional massage practitioner independently. This massage robot is characterized by strong professionalism and high precision, whereas the system requires external support staff for massage positioning. Accordingly, this positioning model runs counter to the goal of integrating massage robots into daily lives. In brief, current massage positioning systems are always dependent on external conditions (e.g., massage manipulation boards and professional doctors) and are not intelligent. Accordingly, understanding the natural way in which people express themselves in the massage area can help the user disengage from the above external dependencies.

It is generally known that the ability to express intentions through physical movements is the most basic and common ability among people [1]. It has been found that when people express something or an area, they usually use gestures or words to direct the attention of others to the target, thus enabling them to gain insights into their intentions [2]. In the case of gestures, people usually use pointing actions to express the target when they are far away from it, that is, indicating behavior [3], which is commonly achieved by extending the index finger and flexing the rest of the fingers [4]. If the target is close, people usually express it in a contact manner, for example, by holding or touching it directly with their hand. Likewise, the above results can be applied to people's representations of the massage area. People typically use static pointing expressions for areas of the body that are distant from the hand. For closer areas, on the other hand, direct contact with the fingertips of the index finger is generally used for expression. On that basis, pointing gestures have become one of the most natural ways of expressing the massage area, and verbal expressions are also one of the most natural ways. Thus, a correct understanding of the above natural expressions can help people disengage from the operating board and reduce memory and operational load. Moreover, people's negative attitudes toward robots can be reduced.

Furthermore, unlike professional massage, daily home massage is characterized by nonspecialist positioning and an unspecified range of massage. As such, autonomous massage positioning faces numerous unique challenges: (1) the system should track information on key points of the human skeleton in real-time, such as the shoulders and waist, as well as hands, to enable massage tracking and (2) the system should identify massage zones and massage points based on an understanding of people's natural expressions.

Accordingly, to solve the above application pain points of intelligent robots, this study focuses on the vital issue of massage area positioning and proposes a method based on natural human-robot interaction with online learning capability.

## 2. Related Work

### 2.1. Positioning of Acupuncture Points

Existing research on massage localization has focused on the identification of body acupoints, and localization is primarily achieved using two methods, including manual-assisted finding and neural network training. The first type of manual assistance requires the marking of the target acupuncture point before the massage, mainly through the posting of the colored origin or 2D codes, after which the system locates the point by identifying the location of the marked point [5, 6]. The manually assisted methods all require a prior manual setting of the reference point and are both less intelligent. The second method, requiring the use of deep learning, is progressively becoming the focus of relevant research. Xiangping and Yudan [7] adopted a neural network model based on particle swarm optimization to train a predictive model of the relative coordinates of acupoints. Later, Sun et al. [8] located two acupuncture points on the human arm with more accuracy using a deep convolutional neural network. Chen et al. [9] used migration learning to transfer the learned facial landmark location network to the acupoint localization network, so as to further increase the accuracy of acupoint localization. The incorporation of location accuracy metrics further increased the accuracy of positioning. The above methods have all produced satisfactory results, whereas the positioning of specific acupuncture points requires professional guidance and planning to achieve the desired results. These methods are contrast to the goal of home-based daily massage, which is primarily aimed at relaxing certain tired areas and does not exert a therapeutic effect. Thus, it is important for intelligent massage positioning systems to understand people's intentions and needs through their behavior.

### 2.2. Intent Understanding with Natural Interaction

Natural human-computer interaction aims to eliminate the boundaries between humans and machines to achieve smooth and natural communication between humans and computers. As research progresses, HCI tends to evolve from the initial passive interaction (e.g., command line interaction and graphical interface interaction) toward active interaction (e.g., machines actively sensing and predicting people's behavior and inferring the user's mental intent) [10, 11]. Human-computer interaction research is committed to achieving intelligent applications. To achieve this goal, a wide variety of sensors are adopted to observe people's physical behavior; human expressions, gestures, gazes [12–14], and other behaviors have also been analyzed in depth. The massage positioning of an intelligent daily massage robot is primarily dependent on the operator's intention, which can be expressed in various ways (e.g., pointing, speech, and gesture). Accordingly, the above modalities need to be considered together to analyze human intentions using contextual information [15–17]. In addition, Liu et al. [18] proposed a multitask model combining STGCN-LSTM and YOLO to recognize human intentions. Batzianoulis et al. [19] proposed the idea of determining control attribution based on people's personal preferences. Kim et al. [20] have proposed a method to identify patterns in people's daily lives that combines intention and event algorithms. Duncan K et al. [21] proposed a Markov model based on a “goal-action-intention network” through iterative Bayesian updating of the network to give it the ability to learn people's habits. Inspired by the above studies, this study adopts a recursive Bayesian algorithm to equip the system with the ability to learn.

### 2.3. Intent Understanding with Natural Interaction

To accurately identify finger-pointing, Smari and Salim Bouhlel [22] implemented fingertip tracking and recognition by contour detection on Kinect depth maps. Shukla et al. [23] proposed an appearance-based probabilistic target detection framework that enables the recognition of pointing gestures and the estimation of pointing directions. Barbed et al. [24] proposed a fine-grained variation of long-range pointing behavior detection using network training. However, it is not possible to obtain highly accurate, real-time finger-pointing information using the above methods. Thus, the focus of research has gradually shifted to the recognition of key points on the body and in the hands. Although Kinect can acquire human skeletal points, it cannot be adopted for accurate pointing since it can acquire a small amount of key information. Simon et al. [25] developed a method to obtain a finger-pointing fine-grained detector through training with a multicamera system to achieve high accuracy in hand keypoint detection. Zhang et al. [26] built a multihand tracking system capable of running on the device in real time and achieving a high degree of accuracy.

In brief, existing massage systems suffer from the above key problems: (1) the system requires auxiliary conditions for manual massage positioning of massage points; (2) the system is unable to learn the massage habits of the user autonomously; and (3) the system is unable to achieve massage at any specific location. In this study, the above key scientific problems are solved by placing a focus on a multimodal intent fusion understanding approach. Combining natural pointing and speech representation, the major elements of intelligent massage systems are investigated (e.g., precise positioning and natural human-machine interaction).

## 3. Materials and Methods

The interaction device of the intelligent massage positioning system primarily comprises a xArm robotic arm, a Kinect perception device, a voice input device, and a computing and processing device, as illustrated in Figure 1. The difficulty of the implementation of the massage positioning system lies in how the system is capable of naturally and accurately sensing the location of the massage area expressed by people with the use of natural pointing gestures and speech. This study proposes an online learning massage positioning algorithm to solve the above difficulty. First, the idea of redundancy is used to extend the intersection of the pointing line and the body into a pointing intersection line to determine a massage candidate area. Second, an interrogative interaction is performed for the massage candidate area using roulette selection to determine the massage center point and the massage point generation model. Lastly, according to the massage area and center point, the selection probability and the central probability of the respective zone under the part are updated. After multiple selections of the same part, the system is capable of learning people's massage habits on the part, thus decreasing the number of interrogation interactions for the next center point confirmation.

To gain insights into the user's intention expressed through speech, a speech intention database, KWLib, should be first created, which describes the correlation between speech and possible intentions. The system uses real-time keyword detection for speech recognition and intent matching. In addition, to understand the user's pointing information, this system detects key points on the body and hands in real-time to achieve pointing recognition. For the intelligent massage positioning system in this study, the two modalities of speech and pointing can be either parallel inputs or single inputs. The input is assigned to three cases: the first is two modalities for parallel input, when it is necessary to determine whether there is a contradiction between the information transmitted by both; if there is, the system will actively remind the user and ask him to re-express it. The second is when two modalities are inputted in parallel, and there is no contradiction identified between them, or only pointing serves as a single modal input. As a result, the system will turn on the OLMP algorithm to massage the localization function. Third, with voice only as the single input, the system will perform a full-area massage on the body part expressed by voice.

Pointing expressions can fall into two types, including contact and noncontact. For the first type of contact expression, the system directly employs the contact point as the center point of the massage. The understanding of the second type of noncontact expression is the difficulty and focus of this study's research. Theoretically, the intersection of the pointing line and the body can be used as the center point of the massage area. However, inaccurate detection of the skeletal points of the body and the user's own reasons (e.g., inability to raise the arm) can cause greater disturbance to the position of the intersection point. Hence, there is an error in using the intersection point as the center point of the massage. It is noteworthy that if the hand is far from the target area, a small deviation in pointing may cause the intersection point to be far from the target point. Furthermore, intelligent massage positioning requires the identification of a massage area rather than just a massage center point. The intelligent massage positioning system proposed is capable of solving the above problems of noncontact expression, and its structure is illustrated in the following diagram:

The system structure consists of three main parts (Figure 2). The first part is the area of number. 1: Through the user's basic input data to understand the intention, to determine the range of the massage candidate area, its main goal is to select a general massage area and reduce positioning errors; the second part is the area of number. 2: Through the roulette selection method to determine the interrogation point within the massage candidate area, its main goal is to determine the location of the massage center point, massage point two-dimensional (2D) distribution model, and massage The third part is the area of number. 3: Based on the user's selection results, the selection probability and central probability of the relevant body parts are constantly updated, and its main aim is to reduce the number of human-computer interactions when positioning the massage center point. The main three sections are elucidated below.

### 3.1. Voice Detection to Determine the Massage Part

We first build a voice intent database KWLib, which stores the set pairs of voice keywords and body part numbers. In addition to body part keywords, the system also focuses on directional words as well as negative words. Finally, all the obtained keyword information is used as the input of the intent database.

Among them, for speech recognition, we use the speech recognition technology of Baidu API to perform real-time speech detection. After the system performs the massage positioning scenario, the system detects the user's voice expression in real time. When the body part keyword is detected, the final body part number is obtained by combining the before and after information. The identification process is shown in Figure 3.

### 3.2. Natural Pointing to Identify Candidate Area for Massage

After considering accuracy, stability, and real time, this study uses the research results of Zhang F et al. and Bazarevsky et al. [27] on hand and body key points as the method of acquiring the base data. The underlying data are processed to identify the candidate area.

First, it is considered that there may be irregularities in user pointing gestures. To increase accuracy, pointing is assigned to two cases. The first case is when the index finger is bent during the pointing process; the second case is when the index finger is not bent during the pointing process. The system sets different pointing lines in accordance with the different cases.

Second, once the pointing line, Line_1_, has been determined, we assume that there exists a surface *α*. The straight line, Line_1_, lies within *α* and that *α* is perpendicular to the ground (the xoz face in 3D space). This study translates the above explicit conditions into mathematical form: the normal **n** of the ground is known to be $\left(\begin{array}{ccc} 0 & 1 & 0 \end{array}\right)$ and let the direction vector **l**_1_ of the line, Line_1_, be $\left(\begin{array}{ccc} a & b & c \end{array}\right)$. With geometric knowledge, the normal vector **n**_*α*_ of the surface *α* is expressed as follows:

(1) $$\begin{array}{c} n_{\alpha }=n\times l_{1}=\left|\begin{array}{ccc} i & j & k\\ 0 & 1 & 0\\ a & b & c \end{array}\right|. \end{array}$$

The equation of surface *α* is obtained by combining the normal vector **n**_*α*_ and the coordinates of the fingertip point. Afterward, the body plane *α*_body_ is obtained from the information on the coordinates of the key points pointing to the body part where the intersection point *p*_intersection_ is located.

Lastly, the length and width of surface *α* and surface *α*_body_ are defined by the position of the pointing hand, the direction of pointing, and the body posture. Afterward, the intersection line *I* between the two surfaces can be found setting the height of the massage candidate area *T* to the length *H* of the projection of *I* on the *y*-axis.

When the user's pointing action is not standard, the system uses the second finger node and the tip of the index finger as the key points of the pointing line, as shown in Figure 4(a). However, when the user's pointing action is standard, the system uses the heel and tip of the index finger as the key points of the pointing line, as presented in Figure 4(b). The red dotted line in the diagram represents the intersection line *I* of the two faces.

The width of the area *T* is obtained by *d* that changes with the distance *d*_*j*_ between the fingertip and *p*_intersection_. If the fingertip is farther away from *p*_intersection_, the intersection point determined by pointing may deviate significantly from the actual target point. Thus, the width of the candidate area *T* should be widened to maximally include the target point within it. Through extensive experimental testing, this study sets the value of *d* for three cases: first is 2 cm < *d*_*j*_ < 8 cm; that is, the distance between the fingertip and *p*_intersection_ is relatively close, and *d* is set to one quarter of the maximum value *L*_1_ of the width of the part where *p*_intersection_ is located; second is 8 cm < *d*_*j*_ < 20 cm, where *d* is set to (1/3)*L*_1_; third is *d*_*j*_ >20 cm; that is, the distance between the fingertip and *p*_intersection_ is relatively far, and *d* is set to (2/3)*L*_1_. Afterward, the length of the projection of *d* and *I* on the *x*-axis is compared, and the maximum value is selected as the width *L* of *T*. The area framed by the dashed line in Figure 5(a) is the candidate area *T*, and the black line within this area is the intersection line *I*.

### 3.3. Determination of Massage Center Point and Massage Point Generation Model in Candidate Area

The results and discussion may be presented separately, or in one combined section, and may optionally be divided into headed subsections.

Before the system was run, this thesis first divided the body into parts, such as the left and right arms, and the back. Second, the respective part was then divided into more refined zones. The respective small zone has a selection probability value and a central probability value, and both two probabilities of the respective small zone under the same part sum to 1. The following is an example of area *T* falling on the back, assuming that the back contains a total of 9 small zones. Then, the determination of the massage point centroid and the massage point generation model is shown below.

Suppose the area *T* contains a total of *m* sections with area values of *S*_1_, *S*_2_... *S*_*m*_, thus forming the set of areas **S**. The selection and central probabilities are obtained for the respective part, resulting in a probability set *θ* and a probability set *μ*, as shown in Figure 5(b). Taking into account the existence of user pointing bias and to avoid the smaller combined probability sections being simply ignored, this study used the roulette selection method to determine the preferred interrogation points within area *T*.

First, the system determines the combined probability for the respective section in area T according to (2) and calculates the cumulative probability value *Q*(*P*_*i*_) for the respective section in order. The cumulative probability for the respective section is the sum of its own probability and the probabilities of all sections that lie before it. The cumulative probability uses line segments of different lengths to represent the probability of the respective section. All sections are integrated to form a long line of length 1.

(2) $$\begin{array}{c} P\left({\text{PT}}_{i}\right)=\frac{S_{i}\times \theta_{i}\times \mu_{i}}{\sum_{j=0}^{m}S_{j}\times \theta_{j}\times \mu_{j}}. \end{array}$$

Next, the system generates a random number in the interval [0,1]. The number is judged to fall within which line segment, so the preferred section of the area T is determined. Notably, the probability of a random number falling in a longer line segment is relatively high. However, there is also the possibility of shorter line segments being selected. Thus, the phenomenon of a fixed range of massage center points is avoided.

The above steps lead to the preferred interrogation section and the position of its center (*x*′, *y*′) within the area *T*. Afterward, the massage arm moves to this center point and asks the user “whether the point currently touched is included in the massage area.” If the system gets a negative answer, the preferred interrogation part will be removed from the candidate area *T*, and the remaining sections will be used as a new candidate area *T*′. The system will then recalculate the combined probability value for the respective section of the area *T*′ and use the above steps to reselect the next section. If a positive answer is obtained from the user, the point (*x*′, *y*′) is moved on the *x*-axis to the intersection line *I* to get a new point (*x*_0_, *y*_0_), and the point serves as the massage center point, as presented in Figure 5(c). In addition, the system sets a minimum area value *β* for the candidate area. When the candidate area is being narrowed down, if the area of the *T*′ is smaller than *β*, the system will ask the user to re-express it.

Lastly, the position coordinates of the massage points are set to be consistent with a normal distribution on the *X* and *Y* axes, and the parameters *x* and *y* are independent of each other. *x*_0_ and *y*_0_ are the means of the two normal distributions, respectively, and the variances are determined by *L* and *H*, respectively. In accordance with the 3*σ* principle, the variance of *X* and *Y* can be found as *σ*_*x*_=(*L*/6) and *σ*_*y*_=(*H*/6), respectively. Accordingly, the equation for the 2D normal distribution that the massage point coordinates obey is expressed as follows:

(3) $$\begin{array}{c} f\left(x,y\right)=\frac{1}{2\pi \sigma_{x}\sigma_{y}}\text{exp}\left(-\frac{x-x_{0}^{2}}{\sigma_{x}^{2}}-\frac{y-y_{0}^{2}}{\sigma_{y}^{2}}\right). \end{array}$$

The system is capable of generating the coordinates of the massage points randomly according to equation (3). In addition, the area enclosed by the four points *x*_0_ − 2*σ*_*x*_, *x*_0_+2*σ*_*x*_, *y*_0_ − 2*σ*_*y*_, and *y*_0_+2*σ*_*y*_ is set as the target area *T*_*t*_ for this massage positioning, as shown in the area framed by the dashed line in Figure 6.

### 3.4. Updating the Central and Selection Probabilities Using Recursive Bayes

To make the results of intention understanding more accurate, the system should be able to learn continuously. In the case of massage positioning, intelligence means that after a number of positions, the system should learn the operator's preferences to achieve more accurate and rapid positioning. To achieve this, this study requires that the system learn the user's historical massage area and massage frequency and be able to automatically update the selection probability values and the central probability values for each small zone under the relevant part. The above goal can be achieved using a recursive Bayesian approach. Suppose that the Rth part of the body is selected *N* times and that the part covers a total of *K* small zones. The result *x*_*R*_^*i*^ of the ith selected massage positioning is expressed as *x*_*R*_^*i*^=(*Q*_*R*1_=0, *Q*_*R*2_=0,…, *Q*_*Ri*_=1,…, *Q*_RK_=0), with *Q*_*Ri*_ representing the ith small zone under the *R*th part. A value of 0 for *Q*_*Ri*_ means that the central point of massage does not fall in the *i*th small zone; a value of 1 for *Q*_*Ri*_ means that the central point of massage falls in the ith small zone. In addition, each of the *K* small zones has a central probability value and a selection probability value, which can form the probability set *θ*_**R**_={*P*_*R*1−center_, *P*_*R*2−center_,…, *P*_RK−center_} and *μ*_**R**_={*P*_*R*1−selection_,…, *P*_RK−selection_}.

Online learning aims to update the central and selection probabilities of the respective small zone under the relevant part using the results of the user's massage positioning selection, that is, to update the probability set *θ*_**R**_ and *μ*_**R**_.

Using Bayes' formula, the posterior probability of the central probability can be written as follows:

(4) $$\begin{array}{c} P\left(\theta_{R}|x^{i}\right)\propto P\left(x^{i}|\theta_{R}\right)\cdot P\left(\theta_{R}|x^{i-1}\right). \end{array}$$

According to (4), the system is capable of understanding user preferences based on continuous learning. The prior function *P*(*θ*_*R*_*|x*^*i*−1^) can be obtained by iterating step by step through *P*(*θ*_*R*_*|x*^*i*−2^),..., *P*(*θ*_*R*_*|x*^0^), that is, *P*(*θ*_*R*_). *P*(*θ*_*R*_) is the initial probability distribution for the small zone. We set it to obey the Dirichlet distribution, and hence, the posterior probabilities also obey the Dirichlet distribution. The likelihood function *P*(*x*^*i*^*|θ*_*R*_) can be obtained by the following equation:

(5) $$\begin{array}{c} P\left(x^{i}|\theta_{R}\right)=\prod_{j=1}^{K}P\left(x_{j}^{i}|\theta_{R}\right)\propto \overset{K}{\underset{j}{\prod }}\theta_{Rj}^{Q_{Rj}}. \end{array}$$

Hence, the maximum a posterior estimate of *θ*_*R*_ is given by the statistically large amount of positioning data, as shown in the following equation:

(6) $$\begin{array}{c} \hat{\theta_{Rj}}=\frac{Q_{Rj}+\alpha_{Rj}-1}{\sum_{i=1}^{K}Q_{Ri}+\sum_{i=1}^{K}\left(\alpha_{Rj}-1\right)}, \end{array}$$

where *α*_*Rj*_ is a Dirichlet parameter that records the prior counts of the observed massage centroids falling in the *j*th zone.

Finally, the selection probabilities are progressively updated according to the way the central probabilities are updated, as shown in the following equation.

(7) $$\begin{array}{c} \hat{\mu_{Rj}}=\frac{C_{Rj}+{\text{HS}}_{Rj}+s_{Rj}}{\sum_{i=1}^{K}C_{Ri}+\sum_{i=1}^{K}{\text{HS}}_{Ri}+\sum_{i=1}^{K}s_{Ri}}, \end{array}$$

where *HS*_*Rj*_ denotes the sum of the areas of the jth small zone contained within the target area of the historical massage; *C*_*Rj*_ represents the area of the jth small zone contained within the current target massage area; and *s*_*Rj*_ is the area of the jth small zone. Thus, the selection probability value *μ*_*Rj*_ for the respective small zone on the *R*th part will be progressively updated as an increasing amount of interaction information is added.

### 3.5. Online Learning Massage Positioning Algorithm

Based on the above discussion, the basic idea of the online learning massage positioning algorithm (OLMP) is elucidated below. (1) When the system detects the noncontact pointing gesture, it exploits the redundancy idea to extend the pointing intersection as the intersection line to determine the massage candidate area T. (2) The system determines the massage center point using the roulette selection method and then determines the 2D normal distribution model of the massage point in accordance with the height and width of the area T. (3) In accordance with the massage target area, the selection and central probabilities of relevant body parts are updated to progressively realize the function of learning the user's massage habit. The algorithm in this study is defined as Algorithm 1.

### 3.6. Algorithm Analysis

The main features exhibited by the OLMP algorithm are elucidated below. (1) The OLMP algorithm can understand the user's representation of any body's position under natural pointing. The system determines the user's pointing direction in accordance with the key point of the finger. If the pointing line does not intersect with the body (e.g., the pointing line points to the outside of the body), the system will actively remind the user and ask him/her to re-express it. If there is an intersection between the pointing line and the body, the system will be consistent with the steps in Section 3.1 to find the candidate area T and determine the center point of the massage within the area T according to Section 3.2. During the above process, the system records the position of the massage point in relation to the body's key points. All the above settings ensure that the massage point is always found when the pointing information is correct. (2) The selection and central probabilities of the respective zone under the body part can be constantly updated online to learn the user's massage habits.

The main differences between the OLMP algorithm and existing methods are elucidated below. (1) The algorithm is capable of achieving massage localization without the need for other auxiliary conditions by analyzing the user's noncontact pointing expression of the massage area under natural conditions. The above function reduces the user's memory and operational load. (2) The algorithm can update the probability value of the respective small zone under the relevant part based on the target area obtained from the localization. This function allows the system to find the massage center point from the massage candidate area T more rapidly in the next positioning, reducing the number of times the system asks the user. (3) In the positioning process, the user can move his body as he pleases without being restricted to a single posture. The above system will achieve real-time tracking of the massage points based on the recorded location of the massage area points in relation to the key points of the body.

## 4. Experimental Results and Analysis

The proposed OLMP algorithm is integrated with the xArm robotic arm for intelligent massage positioning. In this section, the effectiveness and reliability of this proto-type system are further verified, and the intention understanding rate and cognitive load of the algorithm are evaluated.

### 4.1. Experimental Settings

The intelligent positioning system in this study comprises a Kinect device, a computer with an I7-10875H CPU, an RTX2060 GPU, 16G of RAM, and the xArm 7-axis robotic arm. To be specific, the arm was fixed to the table, and the Kinect camera was fixed to the right of the arm, which was approximately 1.2 m away from the user. 20 volunteers between the ages of 35 and 65 were invited to the experiment at a male to female ratio of 1 : 1.

Since the massage arm has a limited range of movement, to achieve effective massage positioning, the area in which the user intends to express himself should be limited, and the user should choose the posture in which the massage can be performed. Moreover, due to the difficulty of expressing the back area by pointing, a special condition was set; that is, the experimenter could point to the front chest, instead of pointing to the back area, and the system would automatically map the front area to the back. However, the experimenter should first verbalize the part of the body that he or she wants to massage. Indeed, the experimenter can also express his or her intention directly to an area of the back.

Furthermore, the types of user responses are classified into positive and negative responses. The keywords of positive responses consist of “yes,” “right,” “correct,” and others, while the keywords of negative responses comprise “no,” “not in,” “negative,” “none,” etc.

### 4.2. Experimental Procedure

The respective experimenter should perform 20 repetitive massage area selections with natural pointing. When the experimenter enters the designated area to express their intention using pointing, if there is a problem with their pointing (e.g., pointing in a direction unrelated to their body), or if there is a contradiction in the parallel input of speech and pointing, the experimenter is asked to repeat the expression, and no count is made in either case. The experimenter can point in a variety of postures (e.g., standing and sitting), as illustrated in Figure 7. If the experimenter is in an area that is out of reach of the robotic arm, the system will alert the user to make position adjustments.

Figure 8 illustrates the whole process of massage localization. Once the pointing gesture is detected and the body posture is stable, the system will determine the candidate area T, which has a height of 200 pixels and a width of 110 pixels, as shown in Figure 8(a). To prevent the body from moving, the system records the position relationship between the massage candidate area points and the rest of the body's key points. Afterward, the OLMP algorithm is used to detect which parts of the area T contain small zones and to determine the preferred interrogation point, as shown in Figure 8(b). The robotic arm moves to this point and initiates the interrogation: does this contact location fall within the target area, as shown in Figure 8(c). When an affirmative answer from the user is detected, the point is moved to the intersection line to obtain the massage center point, and a 2D distribution model of the massage point coordinates is obtained according to equation (3) as follows:

(8) $$\begin{array}{c} \left(x,y\right)=\frac{9}{11000\pi }\text{exp}\left(-\frac{9{\left(x-574\right)}^{2}}{3025}-\frac{9{\left(y-394\right)}^{2}}{10000}\right). \end{array}$$

The system determines the massage target area and the set of massage points based on the 2D distribution model above, as shown in Figure 8(d), and records the location of the massage points in relation to key points on the body. Ultimately, the probability values for the selection and the central of the respective small zone under the relevant part are updated during the positioning process, the experimenter can move or change posture, and the system can achieve real-time tracking of the massage.

### 4.3. Experimental Results

In this study, the proposed OLMP algorithm was validated and evaluated in terms of three metrics, including accuracy, number of interactions, and user cognitive load.

### 4.4. Accuracy

The accuracy of massage positioning can be derived by the following equation:

(9) $$\begin{array}{c} \text{Accuracy Rate}=\frac{\text{Count}}{20}, \end{array}$$

where Count denotes the number of correct massage points in the set **p** of massage points. The counting method is that the robot arm moves to the position of the massage point in **p**, respectively, and asks: “Is the current contact point located in the area you want to massage.” If the answer is positive, the count of Count increases by 1. Otherwise, the count of does not increase.

The results were recorded for 20 experimenters' 20 localization massages, that is, 400 times of intention understanding. The accuracy rate under 400 selections was counted, and the results are presented in Figure 9.

As depicted in the figure, 291 out of 400 intention comprehension tasks achieved a correct rate of 70% or more, for a total of 72.5%. In addition, the cases where the correct rate was below were counted and analyzed, and it was found that the case mainly occurred when the user points directly at the back area with their finger. Due to the limitations of people's limb range of movement, the experimenter's pointing direction and the target area can deviate significantly. The above phenomenon decreases the correct rate of intention understanding.

### 4.5. Number of Interactions

The main innovation of the OLMP algorithm is that the system is capable of learning the user's massage preferences online and decreasing the number of queries for the next massage positioning.

To verify the effectiveness of this innovation, two volunteers were randomly selected and asked to make ten repeatable choices for their back and waist distributions, and the choices should meet their massage needs. To avoid interfering between choices, the experimenter was asked to rest for 10 min after the respective selection was made. When the experimenter is changed, the system resets the initial probability values for the respective area to learn the user's massage habits more rapidly. Furthermore, the system is set to contain 16 small zones on the back of the body and 9 small zones on the waist.

The number of interactions in Figure 10(a)–10(c) implies the number of times the system controlled the robot arm to move to the target point to initiate a query to the user when the center point of the massage within T is being determined. As revealed by the graphs, both experimenters performed a relatively high number of interrogation interactions during the first positioning process. With the increase in the number of times the experimenter positioned the same part, the number of interrogations required decreased. The average number of interactions (c) suggested that after six selections, only one interrogation interaction was generally required to locate the center of the massage. For the random selection model, the number of interrogation interactions does not decrease with the increase in the number of experimenter orientations. Thus, the OLMP algorithm can decrease the number of human-machine interactions during the positioning process by learning the user's massage habits online.

### 4.6. NASA-TLX User Reviews

All 20 experimenters were invited to complete a NASA Task Load Index questionnaire after the experiment was performed. The questionnaire consisted of six evaluation indicators below, including time demand (TD): the efficiency with which time is man-aged during the experiment; physical demand (PD): the level of physical effort demanded by the experiment; personal performance (OP): the level of self-satisfaction in completing the experiment; energy (E): the amount of effort required to achieve the self-assessed level; and frustration (F): how you feel throughout the experiment.

The NASA-TLX generally comprises two steps. Step 1: a two-by-two comparison of the six indicators in 15 sets. The experimenters were allowed to weigh in and select one indicator at a time to calculate the relevance of the indicators to the task. The results are illustrated in Figure 6 as data widths. Step 2: the respective indicator was scored, where the respective indicator was divided into 5 equal intervals, the respective in increments of 1, with 5 as the maximum. The mean values of the correlations between the factors in the 20 questionnaires were derived, as well as the mean value of the respective factor score. The mean variance was obtained as 0.9 for the mental factor, 0.592 for the physical factor, 0.943 for the time factor, 0.843 for the satisfaction factor, 1.122 for the energy factor, and 0.81 for the frustration factor, as illustrated in Figure 11.

As revealed by the statistical results, the OP factor has the highest effect. On the basis of the above factor, the OLMP algorithm is slightly better than the positioning mode of the massager. This finding can be explained below. Since massage chairs have a relatively fixed massage area, they are not sufficiently flexible to target a small area in accordance with the user's wishes. However, the positioning of the massage under natural pointing can be more consistent with the psychological needs of the user, so the OLMP algorithm can bring a higher level of satisfaction to the user. Moreover, as depicted in the graph, the natural pointing and voice expressions carry less load than the operating panel or the remote control. Lastly, a weighted calculation of the six factors gives a total load value of 1.92 for the OLMP algorithm positioning and 2.00 for the massage chair positioning. In brief, the OLMP algorithm positioning has better application prospects than the operator board positioning and also illustrates the effectiveness of the OLMP algorithm. Furthermore, in this study, the age-segmented statistics of the questionnaire was analyzed, and it was found that the OLMP algorithm positioning was much more favorably received by the elderly than the massage chair positioning in terms of the mental factor and the self-satisfaction factor, while the young people's evaluation of the two methods was mixed. As revealed by the above analysis, the OLMP algorithm's core concept can be integrated into elderly assistance and escort robots for intelligent applications.

## 5. Conclusions

In this study, existing massage positioning methods are analyzed, and the OLMP algorithm is proposed by combining the concepts of natural interaction and precise positioning. The OLMP algorithm is to essentially integrate iterative Bayesian online learning of people's daily massage habits for accurate positioning of the massage area with a small amount of interaction. As revealed by the results of the experiments, massage positioning based on the OLMP algorithm can be achieved naturally and in real time without the need for any auxiliary tools and can reduce the memory and operational load on people.

## Figures and Tables

**Figure 1:** Interactive device diagram for intelligent massage positioning systems: (a) Kinect 2.0 devices; (b) xArm robotic arm devices.

**Figure 2:** Illustration of the structure of the massage positioning system.

**Figure 3:** Schematic diagram of the speech recognition process.

**Figure 4:** Intersection line finding diagram with different pointing lines: (a) irregular pointing; (b) regular pointing.

**Figure 5:** Schematic diagram of the massage center point determination process: (a) the area framed by the dotted line represents  *T*; (b) the area, central probability, and selection probability corresponding to each small section contained in the area *T* is indicated; (c) the massage center point is found by moving the interrogation point.

**Figure 6:** Schematic diagram of the massage area determination.

**Figure 7:** Collection of massage positioning charts.

**Figure 8:** The massage area determination process: (a) the candidate area T is determined by pointing lines; (b) the area, selection probability, and central probability of the small area contained in area T are found; (c) the robot arm moves to the preferred point determined by Equation (2) and initiates a query to the user; (d) a positive response is obtained from the user, which leads to the determination of the massage area and the massage point.

**Figure 9:** Distribution of correct rates.

**Figure 10:** Collection of experimental results plots for the online learning function: (a) statistical plots of the number of interactions for #1 experimenter for 10 back and lumbar massage orientations, respectively; (b) statistical plots of the number of interactions for #2 experimenter for 10 back and lumbar massage orientations, respectively; (c) change of the number of interrogative interactions required during online learning.

**Figure 11:** NASA-TLX user evaluation graphs: (a) statistical graph of user evaluations for OLMP algorithm positioning; (b) statistical graph of user evaluations for massage chair positioning.

**Algorithm 1:** Online learning massage positioning (OLMP).

## Data Availability

The source code data used to support the findings of this study have not been made available because the source code belongs to laboratory assets, and we cannot open source without authorization.

## References

[1] Granata C., Ibanez A., Bidaud P. (2015). Human activity-understanding: a multilayer approach combining body movements and contextual descriptors analysis. *International Journal of Advanced Robotic Systems*.

[2] Alibali M. W. (2005). Gesture in spatial cognition: expressing, communicating, and thinking about spatial information. *Spatial Cognition and Computation*.

[3] Butterworth G., Itakura S. (2000). How the eyes, head and hand serve definite reference. *British Journal of Developmental Psychology*.

[4] Mayer S., Schwind V., Schweigert R., Henzex N. The effect of offset correction and cursor on mid-air pointing in real and virtual environments.

[5] Sun K., Zhao Q., Yang Z., Xu X. Visual Feedback System for Traditional Chinese Medical Massage Robot.

[6] Lin S., Yi P. (2019). Human acupoint positioning system based on binocular vision. *IOP Conference Series: Materials Science and Engineering*.

[7] Xiangping Y., Yudan W. (2018). Acupoint positioning system based on pso-bp neural network. *Application of Electronic Technique*.

[8] Sun L., Sun S., Fu Y., Zhao X. Acupoint detection based on deep convolutional neural network.

[9] Chen Y., Yang H., Chen D., Chen X. Facial Acupoints Location Using Transfer Learning on Deep Residual Network.

[10] Sandoval E. B., Brandstetter J., Obaid M., Bartneck C. (2016). Reciprocity in human-robot interaction: a quantitative approach through the prisoner’s dilemma and the ultimatum game. *International Journal of Social Robotics*.

[11] Chaminade T., Rosset D., Da Fonseca D. (2012). How do we think machines think? An fMRI study of alleged competition with an artificial intelligence. *Frontiers in Human Neuroscience*.

[12] Fraune M. R., Sherrin S., Šabanović S., Smith E. R. Is Human-robot interaction more competitive between groups than between individuals.

[13] Belkaid M., Kompatsiari K., De Tommaso D., Zablith I., Wykowska A. (2021). Mutual gaze with a robot affects human neural activity and delays decision-making processes. *Science Robotics*.

[14] Hu Z., Zhang Y., Xing Y., Zhao Y., Cao D., Lv C. (2022). Toward human-centered automated driving: a novel spatial-temporal vision transformer-enabled head tracker. *IEEE Vehicular Technology Magazine*.

[15] Graser A., Heyer T., Fotoohi L. (2013). A supportive friend at work: robotic workplace assistance for the disabled. *IEEE Robotics and Automation Magazine*.

[16] Shishehgar M., Kerr D., Blake J. (2019). The effectiveness of various robotic technologies in assisting older adults. *Health Informatics Journal*.

[17] Hu Z., Xing Y., Gu W., Cao D., Lv C. (2022). Driver anomaly quantification for intelligent vehicles: a contrastive learning approach with representation clustering. *IEEE Transactions on Intelligent Vehicles*.

[18] Liu C., Li X., Li Q., Xue Y., Liu H., Gao Y. (2021). Robot recognizing humans intention and interacting with humans based on a multi-task model combining ST-GCN-LSTM model and YOLO model. *Neurocomputing*.

[19] Batzianoulis I., Iwane F., Wei S. (2021). Customizing skills for assistive robotic manipulators, an inverse reinforcement learning approach with error-related potentials. *Communications biology*.

[20] Kim J. M., Jeon M. J., Park H. K., Bae S. H., Bang S. H., Park Y. T. (2019). An approach for recognition of human’s daily living patterns using intention ontology and event calculus. *Expert Systems with Applications*.

[21] Duncan K. Scene-dependent human intention recognition for an assistive robotic system.

[22] Smari K., Salim Bouhlel M. Gesture recognition system and finger tracking with kinect: steps.

[23] Shukla D., Erkent O., Piater J. Probabilistic detection of pointing directions for human-robot interaction.

[24] Barbed O. L., Azagra P., Teixeira L., Chli M., Civera J., Murillo A. J. Fine-grained pointing recognition for natural drone guidance.

[25] Simon T., Joo H., Matthews I., Sheikh Y. Hand keypoint detection in single images using multiview bootstrapping.

[26] Zhang F., Bazarevsky V., Vakunov A. (2020). Mediapipe hands: on-device real-time hand tracking. https://arxiv.org/abs/2006.10214.

[27] Bazarevsky V., Grishchenko I., Raveendran K., Zhu T., Zhang F., Grundmann M. (2020). Blazepose: on-device real-time body pose tracking. https://arxiv.org/abs/2006.10204.

